# Shenhuang Plaster Application Improves Gastrointestinal Motility in Mice with Postoperative Ileus through Intestinal Microbiota

**DOI:** 10.1155/2022/2823315

**Published:** 2022-08-08

**Authors:** Yanan Shi, Xiao Xu, Ting Liu, Rongyun Wang, Jingming Xu, Yujing Wu, Bin Ding, Qiuhua Sun

**Affiliations:** ^1^The College of Nursing, Zhejiang Chinese Medical University, Hangzhou 310053, China; ^2^The First Clinical Medical College, Zhejiang Chinese Medical University, Hangzhou 310053, China; ^3^College of Life Science, Zhejiang Chinese Medical University, Hangzhou 310053, China

## Abstract

Postoperative ileus (POI) is a common surgical complication, and its incidence remains high. Shenhuang Plaster (SHP) is a famous traditional Chinese medicine with a definite curative effect on postoperative intestinal dysfunction; however, the mechanisms involved in these effects are unclear. Accordingly, in this study, we constructed a POI mouse model and used the intestinal flora as the target to explore the regulatory effect of SHP on gastrointestinal motility. The results illustrated that SHP applied at the Shenque acupoint promoted the recovery of gastrointestinal motility, relieved intestinal villus atrophy and basal damage caused by POI, protected the integrity of intestinal tissue morphology, and alleviated the inflammatory response in the intestinal tissue of POI model mice. In addition, we clarified the role of the intestinal flora in the occurrence and development of POI, further evaluated the changes in the intestinal flora in each group of mice, and analysed the regulatory effect of SHP on the intestinal flora in mice with POI. The results suggested that SHP might improve gastrointestinal motility disorder in POI mice by effectively regulating intestinal flora.

## 1. Introduction

Postoperative ileus (POI) is a common complication of abdominal and nonabdominal surgery. It often manifests as various degrees of abdominal pain, abdominal distension, nausea and vomiting, and weakened or disappeared bowel sounds, and it can lead to further complications such as anastomoses and abdominal infections [1]. With the development of rapid rehabilitation surgery in recent years, POI has been considered the core component that affects patients' postoperative recovery because of the prolonged hospitalisation time and increased hospitalisation costs [2]. At present, the pathogenesis of POI is unclear. Hence, there is a lack of clinically effective treatment methods and drugs. The generally applied treatments, such as gastrointestinal decompression, anti-inflammatory rehydration, and additional nutritional supplements, are not effective [3, 4].

Intestinal inflammation is a major factor that induces POI after surgery. Intestinal surgery can induce intestinal myometrial dendritic cells to produce interleukin (IL)-12 and activate M1 macrophages [5], which can release cytokines and inflammatory mediators such as tumour necrosis factor-*α* (TNF-*α*), IL-1*β*, IL-6, and IL-8 and promote the migration of leukocytes to the intestinal muscle layer [6]. It has been elucidated that surgical procedures often induce dysfunction of the intestinal barrier, which could lead to the translocation of microorganisms and variation of their metabolites [7]. Because the occurrence and development of POI are closely related to intestinal microbes and their metabolites [8], the intestinal flora has become a potential target for the treatment of POI.

At present, the intestinal flora is attracting increasing attention as a drug target for disease prevention and treatment, and traditional Chinese medicine has been increasingly recognised to affect host metabolism and function by regulating the intestinal flora. Our previous studies illustrated that the external treatment Shenhuang Plaster (SHP) applied at the Shenque acupoint (CV8) could effectively promote gastrointestinal transmission and reduce inflammation in the small intestinal smooth muscle [9], and it has already been applied clinically to treat POI [10]. In our previous research, UPLC-MS was applied to identify the main effective components of SHP, including emodin, tanshinone, ginsenoside, and magnolol [11]. Meanwhile, we also found some ingredients of SHP, such as rhein and magnolol, in the sera of rabbits with POI [12]. The prebiotic effects of these active ingredients have been elucidated. In detail, some of these components can enhance the abundance of some probiotics, such as lactic acid bacteria and bifidobacteria, and decrease that of opportunistic bacteria such as *Enterococcus* and *Escherichia shigella* [13–15]. Therefore, we speculated that the application of SHP at CV8 could exert an effect on POI by regulating the structure and function of the intestinal flora. In this study, we revealed the bacterial composition in the small intestine of a mouse model of POI, which may provide new ideas for the clinical application of SHP.

## 2. Materials and Methods

### 2.1. Chemical and Biochemical Materials

Paraformaldehyde was purchased from Tianjin Chemical Reagent Research Institute (Tianjin, China). PBS was purchased from Beijing Zhongshan Jinqiao Biotechnology Co., Ltd (Beijing, China). Ammonia was purchased from Hangzhou Changzheng Chemical Plant (Hangzhou, China). Hydrogen peroxide was purchased from Shanghai Yuanda Peroxide Co., Ltd (Shanghai, China). Methanol was purchased from Shanghai Zhenxing Chemical No. 1 Plant (Shanghai, China). Anhydrous ethanol was purchased from Hangzhou Chemical Reagent Co., Ltd (Hangzhou, China). Ethanol (95%) was purchased from Anhui Ante Biochemical Co., Ltd (Suzhou, China). SHP was previously prepared, and the chemical constituents were identified using UPLC-MS/MS [11].

### 2.2. Animal Treatment

C57BL/6 mice (8 weeks old, 18–20 g) were purchased from the Shanghai Laboratory Animal Centre (Shanghai, China) and handled under a specific pathogen-free condition in the animal experimental centre of Zhejiang Chinese Medical University with a strict light/dark cycle (12 h of light), temperature controlled at 20°C, and free access to food and water. All animal experiments were approved by the ethics committee of Zhejiang Chinese Medical University Animal Research Centre (accepted Nr. 10632). All mice were adaptively fed for 1 week to construct a POI model and randomly divided into the control (Ctrl), model (POI), and intervention groups (POI + SHP), with eight mice per group. After the mice were anaesthetised via isoflurane inhalation, the abdomen of each animal was shaved, disinfected, and covered with sterile gauze, and a 2-cm-long incision was made in the middle of the lower abdomen. The cecum and a part of the small intestine were removed and cleaned using saline-soaked cotton balls for 30 s. The small intestine was then returned to the abdominal cavity, dripped with 1 mL of sterile normal saline, and sutured layer-by-layer while paying attention to protect the intestine from ischaemia and necrosis. After the POI model was established, the animals were fed in separate cages, and SHP was applied at CV8 of mice in the POI + SHP group twice a day.

### 2.3. Gastrointestinal Transmission

Mice were fasted for 24 h and intragastrically administered 6.25 mg/mL FITC-labelled dextran 70 kDa (200 *μ*L) via a gastric tube. After 30 min, the mice were anaesthetised and sacrificed, and the entire gastrointestinal tract was immediately removed by laparotomy and divided into 15 segments (stomach, one segment; small intestine, 10 segments; cecum, one segment; and colon, three segments). Each intestinal cavity was rinsed with saline, and an FITC-labelled glucan cleaning solution was collected. After centrifugation at 12,000 rpm for 15 min, the supernatant was collected, and the absorbance at 494 nm was measured. The percentage and geometric mean of absorbance were calculated for each segment. Gastrointestinal transport function was expressed as the geometric mean and percentage distribution of FITC-labelled glucan absorbance in each segment. The percent absorbance was calculated as follows: percent absorbance = absorbance per section/total absorbance × 100. The geometric mean was calculated as follows: geometric mean = Σ (percentage of absorbance per segment × number of segments)/100.

### 2.4. Morphological and Pathological Observation of Intestinal Tissue

At the end of the experiment, the mice were sacrificed via excessive inhalation of carbon dioxide, and the intestinal tissue (colon and ileum) of mice in each group was collected for morphological and immunohistochemical studies. After formaldehyde fixation for 24 h, 10% formalin-fixed tissue was dehydrated using an alcohol/xylene solution concentration gradient. Then, these dehydrated tissues were embedded in paraffin and cut into 4 *μ*m thick slices. These slices were separated into two groups for histological observation and immunohistochemical studies. One group of slices was stained with haematoxylin and eosin (H&E) and observed under a microscope. Moreover, the ileum and colon of each mouse were hybridised with specific antibodies to detect various proteins.

### 2.5. Real-Time PCR

An RNA extraction kit (TRIzol/chloroform method) was used to extract total RNA from intestinal wall tissue according to the manufacturer's instructions (purchased from American Invitrogen Life Technology Co., Ltd., California, USA). The quality and concentration of the separated mRNA were determined by the ratio of absorbance at 260 and 280 nm. The extracted total RNA was quantitatively detected using a NanoDrop (Thermo Fisher Scientific, USA) and then reverse-transcribed into cDNA with SuperScript III (Invitrogen). The cDNA was used as the template for real-time PCR. The PCR protocol consisted of template denaturation at 95°C for 5 min followed by 45 amplification cycles of 95°C for 10 s, 55°C for 30 s, and 72°C for 10 s. The melting curve was monitored as the temperature increased from 65 to 95°C. *β*-actin was used as an internal reference gene. The relative expression of the target gene of each sample was calculated using the 2^−ΔΔCt^ method. The specific primer pairs for target quantification are listed in Table 1.

### 2.6. 16S rRNA Gene Sequencing and Intestinal Flora Characterisation

A faecal DNA extraction kit was used to extract DNA from 200 mg of frozen faeces. The extracted DNA was quantified using a NanoDrop and purified by 1.0% agarose gel electrophoresis. A Phusion Hot Start Flex 2 × Master Mix was used to amplify the V3-V4 regions of the 16S rDNA gene by PCR with a universal primer pair (341F, 5′-CCTACGGGNGGCWGCAG-3′; 805R, 5′- GACTACHVGGGTATCTAATCC-3′) [9]. The sequencing library was constructed, and the Qubit and Agilent 2100 analyzers were used to quantify the library and evaluate the quality of the library. A 275–450-bp insertion sequence was selected for sequencing on the Illumina NovaSeq platform. The low-quality sequences and contaminating sequences from the host were deleted to obtain the clean data. SOAP de novo (v2.04) was used to assemble and analyse clean data. MetaGeneMark was used for gene prediction and nonredundant gene set construction. MyTaxa and related databases were used to obtain the species annotation information of each gene and species abundance tables at different taxonomic levels. Based on the species abundance table and functional abundance table, linear discriminant analysis effect size (LEfSe), principal component analysis (PCA)/principal coordinate analysis, and sample cluster analysis were performed.

### 2.7. Statistical Analysis

In this research, the measurement data were expressed as the mean ± SD, and SPSS 22.0 statistical software was used for analysis and processing. The least significant difference test was used for pairwise comparisons between groups, analysis of variance was used for comparisons of homogeneity of variance among multiple groups, and the Kruskal–Wallis H test was used for comparisons of uneven variance among multiple groups. *P* < 0.05 denotes statistical significance.

## 3. Results

### 3.1. SHP Alleviated POI-Induced Body Weight Loss

The mice in the Ctrl group had a good mental and physical status throughout the experiment, including smooth and shiny hair and normal food consumption. The mice in the POI group were dull and sluggish, they huddled up in the corner, and they rarely ate. After SHP administration, the mental state, activity, glossiness, and food intake of POI mice were improved. Simultaneously, we monitored the body weight of the mice every other day. As presented in Table 2, the weight gain of mice in the POI group was significantly lower than that of mice in the Ctrl group (*P* < 0.001), whereas mice in the POI + SHP group gained significantly more weight than mice in the POI group (*P* < 0.05), suggesting that SHP could effectively restore the food intake and body weight of mice.

### 3.2. SHP Improved POI-Induced Gastrointestinal Motility Dysfunction

The gastrointestinal motility of mice was compared according to the fluorescence of various parts of the gastrointestinal tract. As presented in Figure 1(a), fluorescently labelled dextran (70 kDa) was rapidly transmitted in the Ctrl group, and the greatest fluorescence was detected in SI9 (terminal ileum). In the POI group, fluorescent dextran accumulation was greatest in SI1 (the first segment of the ileum), indicating accumulation at the beginning of the gastrointestinal tract, and the transmission of fluorescence was severely hindered. In the POI + SHP group, fluorescent glucan accumulated in SI8 (ileum) at a significantly faster rate than observed in the POI group and a similar rate as that in the Ctrl group. The geometric mean (geometric centre (GC)) of gastrointestinal transmission in each group is presented in Figure 1(b). The GC values of the Ctrl, POI, and POI + SHP groups were 8.34 ± 0.52, 3.11 ± 0.45, and 6.40 ± 0.30, respectively. Compared with the findings in the Ctrl group, the GC value was significantly lower in the POI group (*P* < 0.001), whereas the value was significantly higher in the POI + SHP group (*P* < 0.001). The aforementioned results fully demonstrated that POI could cause obvious gastrointestinal motility dysfunction, and gastrointestinal transmission function was significantly reduced. The topical application of SHP significantly improved the dysfunction induced by POI.

The length of the villus and thickness of the mucosal layer are the two main intestinal morphological parameters for evaluating intestinal health. Therefore, this study performed H&E staining of the colon and ileum of different mice and measured the villus length and mucosal layer thickness. As presented in Figure 2, the colon and ileum tissues in mice in the Ctrl group were intact, with no obvious oedema, congestion, and obvious inflammatory cell infiltration, and the villus and mucosal layer were intact and undamaged. Extensive inflammatory cell infiltration was observed in the colon and ileum in mice in the POI group, in addition to muscle layer damage in some tissues, intestinal structure disorder, villus and muscle layer damage, villus atrophy and basal damage. The changes in the villus and mucosal layer were significantly different from those in the Ctrl group (*P* < 0.001). The histopathological performance of the colon and ileum in POI + SHP mice was significantly better than that of POI mice, including significantly reduced inflammatory cell infiltration and villus and mucosal layer damage and improved villus length and mucosal layer thickness (*P* < 0.05), suggesting that SHP could improve the morphology and function of intestinal tissue.

The results of immunohistochemistry illustrated that the expression and distribution of cyclooxygenase (COX)-2 protein in the colon and ileum of mice in each group were significantly different (Figure 3(a)). The expression and distribution of COX-2 in the colon and ileum of POI mice were significantly increased (especially the colon), and the positive area was significantly larger than that of Ctrl mice (*P* < 0.001). The expression and distribution of COX-2 were significantly lower in the POI + SHP group than in the POI group, and the positive area (relative value) was significantly lower than that in the POI group (*P* < 0.001). In addition, as presented in Figure 3(b), the expression and distribution of inducible nitric oxide synthase (iNOS) protein, which plays an important role in the formation of nitric oxide (NO), were also significantly different in the colon and ileum among the groups. The expression and distribution of iNOS in the intestinal tissue of mice were significantly higher in the POI group than in the Ctrl group (especially in the colon), and the positive area was significantly larger in the former group (*P* < 0.001). Compared with the results in the POI group, the expression and distribution of iNOS were reduced, and the positive area (relative value) was smaller in the POI + SHP group (colon, *P* < 0.05; ileum, *P* < 0.001). The aforementioned results indicated that SHP could effectively inhibit the expression and distribution of COX-2 and iNOS, thereby inhibiting the inflammatory response of intestinal tissues.

In this study, qRT-PCR was used to detect the mRNA expression of inflammatory mediators (IL-1*β*, IL-6, tumour necrosis factor (TNF)-*α*, T-bet, COX-2, and iNOS) in the smooth muscle of the small intestine tissue. As presented in Figure 3(c), the expression of IL-1*β* (*P* < 0.001), IL-6 (*P* < 0.001), TNF-*α* (*P* < 0.001), T-bet (*P* < 0.01), COX-2 (*P* < 0.001), and iNOS (*P* < 0.001) was significantly higher in the POI group than in the Ctrl group, suggesting that the intestinal tissue of POI model mice had obvious inflammation. After treatment with SHP, the expression of IL-1*β* (*P* < 0.05), IL-6 (*P* < 0.01), TNF-*α* (*P* < 0.001), COX-2 (*P* < 0.001), and iNOS (*P* < 0.01) in the intestinal tissue of mice was significantly decreased, indicating that the topical use of SHP at CV8 could reduce the mRNA expression of inflammatory mediators in the smooth muscle of the small intestine and relieve the intestinal inflammation caused by POI.

### 3.3. SHP Regulated POI-Induced Intestinal Flora Imbalance

In this study, the effect of SHP on intestinal flora was determined by sequencing the V3-V4 regions of 16S rDNA. In total, 20 samples were sequenced (Ctrl group, five samples; POI group, six samples; POI + SHP group, nine samples). A total of 1,422,245 Raw_Tags were obtained. After data processing and filtering, clean data were obtained, and the effective sequence length was 1,140,229. The average effective rate of sequencing data was 80%. The final feature average value was 764, including averages of 997, 506, and 806 in the Ctrl, POI, and POI + SHP groups, respectively. All values met the minimum value required for sequencing.

The alpha diversity analysis results (Figure 4(a)) revealed in the intestinal flora of mice among the groups. POI reduced the alpha diversity in the intestinal flora, including species richness and uniformity, whereas these changes were reversed by SHP supplementation. In this study, the Shannon value was used to represent the richness and uniformity of the species, with higher values indicating greater diversity. The beta diversity analysis results illustrated that in PCA (Figure 4(b)), there was a clear separation among the groups. The samples of the Ctrl and POI groups were distributed separately without any intersection. Six samples in the POI + SHP group were clustered closer to the Ctrl samples, and three samples were clustered with the POI samples. The difference in community composition among the groups was statistically significant (*P* < 0.05).

In terms of the structure and composition of the intestinal flora at the phylum level (Figure 4(c)), the abundance of Bacteroidetes and Firmicutes was highest in the Ctrl group, and their abundance was significantly lower in the POI group. Meanwhile, the abundance of Proteobacteria increased from 4.39% in the Ctrl group to 35.97% in the POI group. The relative abundance of Bacteroidetes and Firmicutes was higher in the POI + SHP group than in the POI group, and the abundance of Proteobacteria decreased to 11.67% in the POI + SHP group. At the genus level (Figure 4(d)), the abundance of Muribaculaceae_unclassified was the highest in the Ctrl group. The relative abundance of the pathogen *Klebsiella* was highest in the POI group, whereas its relative abundance was extremely low in the Ctrl and POI + SHP groups (0.01 and 0.05%, respectively). The abundance of Muribaculaceae_unclassified was significantly lower in the POI group than in the Ctrl group. The abundance of Muribaculaceae_unclassified was higher in the POI + SHP group than in the POI group, whereas that of *Klebsiella* and *Parabacteroides* was significantly lower.

The results of LEfSe (Figure 4(e)) indicated that at the phylum level, Proteobacteria was significantly enriched and Firmicutes was significantly suppressed in the POI group, whereas Firmicutes was significantly enriched and Proteobacteria was significantly depressed in the intestines of mice in the POI + SHP group. At the genus level, pathogenic bacteria, such as *Klebsiella*, *Enterobacter*, and *Enterococcus*, were significantly enriched in the intestinal flora of POI model mice but significantly suppressed in the POI + SHP group. The relative abundance of probiotics such as Lachnospiraceae_NK4A136_group, Eubacterium__xylanophilum_group, *Muribaculum*, Ruminococcus_1, Ruminococcaceae_UCG_014, Ruminiclostridium_6, *Oscillibacter*, and *Paramuribaculum* was significantly decreased in the POI group and significantly enriched in the POI + SHP group.

Correlation analysis of intestinal flora and intestinal function evaluation indices of POI model mice revealed that the enrichment of the intestinal flora in POI model mice had significantly negative correlations with intestinal function evaluation indices (D-value of body weight, GC value, intestinal villus height, and basal thickness). Meanwhile, the enrichment of the intestinal flora in POI model mice was positively correlated with iNOS and COX-2 expression in the colon and ileum. Specific to the flora, the abundance of *Klebsiella* and *Enterococcus* was positively correlated with iNOS and COX-2 expression in the colon, and the abundance of *Enterococcus* was negatively correlated with the GC value, D-value of body weight, and villus height.

## 4. Discussion

POI is a common complication of surgery that seriously affects patients' postoperative recovery, prolongs the treatment cycle, reduces patients' quality of life, and exerts a certain amount of economic pressure on patients' families as well as society [16]. To prepare POI model mice in this study, the small intestine of C57BL/6 mice was wiped with a saline-soaked cotton ball, and the application of SHP at CV8 in POI model mice produced obvious improvements. In detail, the application of SHP at CV8 significantly promoted gastrointestinal transport function in POI mice, reduced the damage of intestinal tissue caused by wiping, and alleviated the inflammatory reaction in intestinal tissue. In addition, SHP significantly reversed the dysbiosis of intestinal flora and protected intestinal homeostasis by increasing the diversity of intestinal flora, promoting the growth of intestinal probiotics, and inhibiting the growth of intestinal pathogens.

In this study, the gastrointestinal transmission capacity and GC value were significantly decreased in POI model mice, highlighting serious damage to gastrointestinal motility, which also verified the feasibility of the POI model in this experiment. This was consistent with previous studies, which suggested that POI mice had serious dysfunction of gastrointestinal transmission [17]. At the same time, the intestine of POI mice displayed severe damage including obvious intestinal villus and basal layer atrophy. Identity to that of our previous studies [11], SHP significantly promoted the recovery of gastrointestinal motility and protected the integrity of intestinal histomorphology in POI mice, and these effects may be attributable to both the effects of the drug and stimulation of the acupoint.

Inflammation of small intestinal smooth muscle is a key factor leading to POI. It has been demonstrated that the release of inflammatory factors in small intestinal smooth muscle is the crucial pathological change of POI [18]. Intestinal macrophages can mediate the inflammatory response, and their dysfunction induces an imbalance of this response. In detail, intestinal injury promotes the activation of macrophages, which release inflammatory mediators such as IL-6, TNF-*α*, IL-1*β*, and T-bet that can induce iNOS and COX-2 expressions. Although some published literature suggests that many ingredients in SHP can reduce the expression of inflammatory mediators in intestinal tissue, the present work initially validated the regulative capability of SHP application on the expression of these proteins, which might be related to the anti-inflammatory effect of its multiple effective components [19, 20]. Actually, physcion can inhibit the release of NO [21]. Aloe–emodin and emodin can suppress the mRNA expression of TNF-*α* [17, 22]. Rhein has good anti-inflammatory effects, and it can alleviate gastrointestinal reactions [23]. And these ingredients in SHP have been previously identified [11].

The intestinal flora is a critical factor influencing the fitness of the intestine and body health, which could be affected by not only food or medicine intake but also massage, acupuncture [24, 25]. Previous studies suggested that the intestinal flora plays a crucial role in wound healing, which is one of the major aetiological factors of POI. It has been commonly recognised that postoperative complications, such as postoperative infection or delayed postoperative intestinal motility disorder, might be related to an imbalance of the intestinal flora [26, 27]. The pathogens, *Klebsiella*, *Enterobacter*, and *Enterococcus*, which were significantly enriched in the intestinal flora of POI mice in our study, highly correlated with many infectious diseases of humans [28, 29]. In addition, expression of iNOS and COX-2 in colon cells has been observed with the enrichment of *Klebsiella* and *Enterococcus*, which had negative correlations with the GC value, D-value of body weight, and intestinal villus height [30]. SHP application selectively inhibited the enrichment of *Enterococcus*, *Klebsiella*, and *Enterobacter*. This result indicated that SHP application on CV8 could also influence the gut microbiota. Unfortunately, the further bio-mechanisms of SHP's efficacy has not been clarified in this study. The published literature suggests that some ingredients, such as emodin, a prebiotic that is beneficial for the growth of lactic acid bacteria and bifidobacteria [13, 31], could be transdermally absorbed. Otherwise, the umbilical application of rhubarb (an ingredient in SHP) can significantly improve the recovery of postoperative bowel and reduce the incidence of postoperative abdominal distension [32]. Magnolol in SHP can improve gastrointestinal qi stagnation and inhibit intestinal muscle spasm [33]. Meanwhile, we hypothesised that these ingredients in SHP were percutaneous absorbed and improved the postoperative recovery and disorder of the immune response of the intestine, as well as the gastrointestinal microflora.

## 5. Conclusion

The intestinal flora plays a key role in the occurrence and development of POI. The external application of SHP at CV8 significantly promoted the recovery of intestinal motility and downregulated the expression of inflammatory mediators in POI model mice, by improving the regeneration of intestinal epithelial cells, inhibiting the intestinal inflammation, and maintaining intestinal immune homeostasis, which might relate to the intestinal flora.

## Figures and Tables

**Figure 1:** Intestinal motility evaluation. (a) Gastrointestinal transmission curves: the distribution of fluorescein-labelled dextran in the gastrointestinal tract (St, stomach; SI, small intestinal segments 1–10; Co, colon segments 1–4) of mice in each group. (b) Derived geometric centre of mice in each group. The significant differences, marked with asterisks, were in comparison with the Ctrl (^*∗∗∗*^*P* < 0.001), and the significant differences, marked with triangles, were in comparison with the POI (^ΔΔΔ^*P* < 0.001). Ctrl, control group; POI, postoperative ileus group; POI + SHP, Shenhuang Plaster-treated POI group. SHP protected the integrity of intestinal morphology.

**Figure 2:** Histological analysis of the intestine. (a) Image of haematoxylin and eosin-stained colon and ileum of Ctrl, POI, and POI + SHP mice. (b) Average length of the intestinal villus and thickness of the mucosal layer in the colon and ileum of mice in each group as measured using NDP view software. The significant differences between the POI and Ctrl groups are indicated with asterisks (^*∗∗∗*^*P* < 0.001), and the significant differences marked with triangles was in comparison between the POI + SHP and the POI groups (^ΔΔΔ^*P* < 0.001). Ctrl, control group; POI, postoperative ileus group; POI + SHP, Shenhuang Plaster-treated POI group. SHP inhibited POI-induced inflammation of intestinal tissue.

**Figure 3:** Measurement of inflammatory responses in intestinal tissue via immunohistochemistry. (a) The expression and distribution of COX-2 protein in the colon and ileum in each group. (b) The expression and distribution of iNOS protein in the colon and ileum in each group. (c) Relative expression of some inflammatory cytokines in the ileum and colon of mice in different groups. Data are presented as fold changes compared with that of the Ctrl group. Differences between the POI and Ctrl groups are indicated by asterisks (^*∗*^*P* < 0.05, ^*∗∗*^*P* < 0.01, ^*∗∗∗*^*P* < 0.001), and differences between the POI + SHP and POI groups are indicated by triangles (^Δ^*P* < 0.05, ^ΔΔ^*P* < 0.01, ^ΔΔΔ^*P* < 0.001). Ctrl, control group; POI, postoperative ileus group; POI + SHP, Shenhuang Plaster-treated POI group; IL, interleukin; TNF, tumour necrosis factor; COX, cyclooxygenase; iNOS, inducible nitric oxide synthase.

**Figure 4:** Changes in the intestinal flora of mice in each group. (a) Analysis of alpha diversity. (b) Analysis of beta diversity. (c) Histogram of the structure and composition of the intestinal flora at the phylum level. (d) Histogram of the structure and composition of the intestinal flora at the genus level. (e) Differential species evolutionary branch diagram of the intestinal flora. (f) Correlation analysis of the intestinal flora and intestinal function evaluation indices of POI model mice. Ctrl, control group; POI, postoperative ileus group; POI + SHP, Shenhuang Plaster-treated POI group.

**Table 1:** Primer sequences.

Target cytokines	Forward (5′ to 3′)	Reverse (5′ to 3′)	Gene loci
IL-1*β*	TCATGGGATGATGATAACCTGCT	CCCATACTTTAGGAAGACACGGATT	Chromosome 2, NC_000068.8 (129206490.129213059, complement)
IL-6	CTTTTGAIATATGGAAT	CCAGTTTGGTAGGCATCCATC	Chromosome 5, NC_000071.7 (30218112.30224973)
Tbx21	CAAGTGGGTGCAGTGTGGAAAG	TGGAGAGACTGCAGGACGATC	Chromosome 11, NC_000077.7 (96988833.97006157, complement)
TNF-*α*	CCCTCACACTCAGATCATCTTC	GTTGGTTGTCTTTGAGATCCAT	Chromosome 17, NC_000083.7 (35418343.35420983, complement)
COX-2	CAACTCTATATTGCTGGAACATGGA	TGGAAGCCTGTGATACTTTCTGTACT	Chromosome 1, NC_000067.7 (149975782.149983985)
iNOS	CAGCTGGGCTGTACAAACCTT	CATTGGAAGTGAAGCGTTTGG	Chromosome 11, NC_000077.7 (78811613..78851052)
*β*-Actin	TTCCAGCGTTCCTTCTTGGGT	GTTGGCATAGAGGTGTTTACG	Chromosome 5, NC_000071.7 (142888870.142892509, complement)

IL, interleukin; TNF, tumour necrosis factor; COX, cyclooxygenase; iNOS, inducible nitric oxide synthase.

**Table 2:** Changes in body weight in each group (g).

Group	Initial weight	Final weight	Body weight gain
Ctrl	21.65 ± 1.47	23.05 ± 1.62	2.23 ± 0.94
POI	22.22 ± 1.53	21.02 ± 1.46	−1.20 ± 0.46^*∗∗∗*^
POI + SHP	21.04 ± 0.66	20.4 ± 0.61	0.64 ± 0.24^△△△^

*Note.* The significant differences, marked with ^*∗*^ and ^Δ^, were compared with that of the Ctrl and POI groups, respectively, in this study. The significant differences between the POI and Ctrl groups are indicated by asterisks (^*∗∗∗*^*P* < 0.001 and ^ΔΔΔ^*P* < 0.001). Ctrl, control group; POI postoperative ileus group; POI + SHP, Shenhuang Plaster-treated POI group.

## Data Availability

All data used to support the findings of this study are included within the article, and these data can also be accessible on website https://fairsharing.org/collection/ShenhuangPlaster Application Improves Gastrointestinal Motility in Mice with Postoperative Ileus through Instestinal Microbiota or requested from the corresponding author of this manuscript (sunqiuhua@zcmu.edu.cn).
